# Analysis of Chinese Machine Translation Training Based on Deep Learning Technology

This article has been retracted.

**DOI:** 10.1155/2022/6502831

**Published:** 2022-08-02

**Authors:** Yiqun Sun

**Affiliations:** College of Foreign Languages, Ocean University of China, Qingdao, China

## Abstract

With the advent of the information age, people can establish good communication through Internet technology. Mechanical translation has become a key means to solve people's communication problems. However, there are still obstacles to communication between different languages. In order to solve this problem, this paper uses existing neural network technology to the English-Chinese bidirectional machine translation model in the field of marine science and technology. Based on deep learning technology, we collect Chinese and English abstracts and partial full texts of Chinese and English papers with marine science and technology as the key words and build a professional corpus in English and Chinese about marine science and technology. In the Chinese-English bidirectional translation model, the local weight sharing is introduced into the Chinese encoder and the English encoder, and the output of the Chinese encoder sublayer and the English encoder sublayer is fused as the output of the respective encoders, and the performance of the translation model is evaluated using the BLEU parameters. Through the training of the translation model, compared with the transformer model, the BLEU value of the model with local weight sharing and encoder sublayer fusion output is improved by 1.6 and 3.8 in the Chinese-English and English-Chinese translation directions, respectively. The PPL values in the Chinese-English and English-Chinese translation directions decreased by 18.72% and 14.62%, respectively. We demonstrate the effectiveness of the language translation model. Experiments show that the research on machine language adaptive technology based on deep learning can more smoothly realize the two-way translation of literature in the field of marine science and technology. Compared with traditional mechanical translation, this paper proposes a translation model based on the deep neural algorithm, which improves the effect of model training by constructing a Chinese-English corpus with the theme of marine science and technology.

## 1. Introduction

According to incomplete statistics, there are now around 7,000 human languages [1]. Most of the current machine translation technology is based on big data. Only by training on a large amount of data can we get a better effect. In fact, only a few languages such as Chinese, English, French, and German have more training data, and there are almost no training resources available for other languages [1]. In some specialized fields, such as marine science and technology, there are fewer resources in Chinese and other languages. On very little data, it is very difficult to train a good system. Around the 1990s, researchers proposed the statistical machine translation (SMT) based on statistical techniques and established a corresponding mathematical model of machine translation [2, 3]. The model can be trained on a large amount of data and is suitable for all languages. Once the model is trained, fast bidirectional translation between two languages can be achieved at very low cost. Statistical machine translation is a corpus-based method. The data in the corpus are small, which will cause the problem of sparse data and affect the training effect of the SMT model, making it difficult to obtain accurate and fluent translation results. At the same time, the question of how to add expert knowledge to the machine translation model is another major challenge faced by machine translation. At present, the knowledge of machine translation comes from automatic training of big data. The knowledge obtained from this training is still far from the knowledge of language experts, thus affecting the effect of machine translation.

With the advent of the era of network science and technology, the situation of mutual integration of the global economy appears. Under this background, promoting the exchange of professionals is an important task of national rejuvenation. With people's attention to the marine, marine science and technology has become a key research and development area for various countries. Although English and Chinese are commonly used languages in the world, there are relatively few studies on Chinese and English corpora related to marine science and technology, especially the lack of high-quality, large-scale parallel corpora, which is not conducive to the mutual translation of marine science and technology literature. Machine translation (MT) was first proposed by the American translation pioneer Warren Weaver in 1949 [4]. It has attracted extensive attention in the world. At that time, due to technical reasons, the texts translated by machine were full of errors, difficult to use, and failed to be popularized and applied, which also made people suspicious of machine translation technology, and its research once fell into a low ebb. Until the 21st century, neural network technology developed rapidly and was successfully used in machine translation technology, making machine translation a breakthrough [5]. Deep learning is currently the most popular and effective neural network learning technology, which uses multiple layers of nonlinear transformations to map high-dimensional abstract expressions. Machine translation based on deep learning technology can achieve fast and accurate translation between two languages, but the premise is that the training of machine translation models requires a large number of parallel corpora. In the research on the English-Chinese translation of marine scientific and technological literature, if we want to achieve a smooth conversion of mechanical language, we should expand the research on the corpus to improve the effect of English-Chinese translation in the field of marine science and technology [6].

In order to improve the training effect of the model, the Chinese-English corpus data with important data significance will be captured from professional literature and a Chinese-English parallel corpus will be constructed for machine training. Based on the transformer model, the idea of local weight sharing and encoder sublayer fusion output is introduced to optimize and improve the translation model and enhance the professional applicability of the language model. The translation model is trained based on the Chinese English parallel corpus. The verification results show that the proposed English-Chinese translation model of marine scientific and technological literature is feasible and can achieve good language conversion.

The innovation of the research is that based on the traditional mechanical translation, a translation model based on depth neural algorithm is proposed and crawls important Chinese English corpus of marine scientific and technological literature to increase the effect of model training. The idea of local weight sharing and encoder sublayer fusion output was introduced to optimize and improve the machine translation model and improve the effect of training. In order to better verify the effect of training, the BLEU value is introduced as the evaluation standard to verify the feasibility of the translation model.

The second part mainly introduces the relevant research and application results of machine translation adaptive technology of deep learning. The third part mainly introduces the summary framework of the marine science and technology Chinese English translation model of the parallel corpus and introduces the local weight sharing and encoder sublayer fusion output to optimize the translation model. The fourth part analyzes the simulation data of the marine science and technology Chinese English translation model and verifies the feasibility of the proposed translation model.

## 2. Related Work

Machine translation (MT) is an important tool for realizing cross-language communication. Machine translation can be roughly divided into dictionary-based machine translation [7], rule-based machine translation [8], statistics-based machine translation [3], and neural network-based machine translation according to the development stage [9].

At present, with the wide application of deep neural networks in natural language processing, machine translation based on neural networks has achieved good performance and has become the mainstream method in the current field of machine translation [9]. Scholars have also conducted a lot of research.

Ye et al. used the word alignment structure of statistical machine translation as external word alignment information and introduced it into the decoding step of neural machine translation to guide the neural machine translation decoder to estimate the target language more accurately. Experimental results show that the data processing method based on language model and sentence similarity can ensure data quality to a certain extent, and the neural machine translation model integrating statistical machine translation vocabulary alignment structure can effectively improve the effect of machine translation [10].

Laskar et al. propose a multimodal corpus suitable for the multimodal translation task of English-Assamese pairs to implement a multimodal neural machine translation model. The comparison of automatic evaluation metrics between text-only and multimodal neural machine translation shows that multimodal neural machine translation outperforms text-only neural machine translation [11].

Zhang proposed a cloud computing-based machine-assisted translation system design for the long translation time of current machine-assisted translation systems. A new machine-aided translation system is designed by referring to the cloud computing model. The hardware of the system is divided into four layers: user layer, service layer, computing layer, and storage layer. The test results show that the translation time of the machine-assisted translation system based on cloud computing is shorter than that of the traditional machine translation system [12].

In order to solve the problem of time-consuming and frequent mistranslation of traditional translation methods, Li and Wang designed an English-Chinese machine translation method based on transfer learning. The experimental results show that the method has short translation time and fewer mistranslations [13].

Zhang et al. propose to introduce explicit phrase alignment in the translation process of the arbitrary neural machine translation model. The key idea is to build a search space similar to that of phrase-based statistical machine translation for neural machine translation where phrase alignment is readily available. Experiments show that the method makes the translation process of neural machine translation more interpretable without sacrificing translation quality, achieving significant improvements in translation tasks where vocabulary and structure are constrained [14].

Sennrich et al. of the University of Edinburgh first applied the back translation method to the field of neural machine translation in 2016, which improved the effect of low-resource translation [15]. The method first uses high-quality parallel sentence pairs to train the initial model, then translates the target monolingual into the source monolingual through the initial translation model, and finally retrains the model by mixing the reverse translated sentence pairs with the original corpus. Subsequently, some scholars studied the effect of the ratio of real data and back-translation data on the translation effect [16] and proposed methods to improve pseudo-parallel corpus [17–19].

Neural machine translation (NMT) has made impressive progress in the past few years, but the language model attribute of NMT tends to produce fluent but sometimes unfaithful translations, which hinders the improvement of translation capacity. In response to this problem, Chen et al. proposed a simple and effective method to integrate prior translation knowledge into NMT in a general manner compatible with neural networks, thereby making full use of the prior translation knowledge to enhance the performance of NMT [20].

Lin team found that the resources of Chinese-English parallel corpus are insufficient and proposed to use deep learning to complete Chinese-English conversion. The research results improve the performance of Chinese-English neural machine translation [21]. Ercan and Haziyev explored the potential of meaning induction in large-scale multilingual translation maps and proposed the performance of the graph clustering method in syntax set detection. The system can produce WordNet from scratch. The coverage of WordNet basic concepts in 51 languages ranges from 20% to 88% and expands the existing WordNet to 30% [22]. Lora et al. proposed a middle encounter method to create a virtual platform of heterogeneous systems and automatically integrate the component model into a single homogeneous system level executable description. Through the analysis of typical design processes, the classification of the design domain/abstraction level is defined [23]. The purpose of Dhanjal and Singh research work is to develop an automatic system to translate speech into Indian sign language using avatar (SISLA). The minimum accuracy of the proposed training model for English, Punjabi, and Hindi is 91%, 89%, and 89%, respectively [24].

The fast advancement in machine translation models necessitates the development of accurate evaluation metrics that would allow researchers to track the progress in text languages. The evaluation of machine translation models is crucial since its results are exploited for improvements of translation models. A detailed classification and comprehensive survey of various fully automated evaluation metrics were conducted by Chauhan and Daniel grouped into five categories, namely, lexical, character, semantic, syntactic, and semantic and syntactic, for better understanding [25].

Liu introduced the automatic machine translation language vector function into the translation quality evaluation model based on deep learning to realize automatic evaluation of machine translation quality [26].

Through the study of relevant data, it can be found that deep learning technology has a wide range of applications, introducing deep learning technology into traditional mechanical translation, constructing marine science and technology Chinese-English mechanical translation model with parallel corpus based on neural network technology, and introducing the idea of local weight sharing and encoder sublayer fusion output to optimize and improve the translation model can effectively improve the accuracy of traditional mechanical translation. It has an important reference value for the current research in the field of mechanical language.

## 3. Construction of the Machine Translation Model Based on Deep Learning

### 3.1. Principles of a Mechanical Translation Model

Machine translation has the advantages of low cost, simple and fast process, and fast translation speed, and can translate large amounts of text in almost real time. At the same time, machine translation can target multiple users and languages at the same time, and you can even translate text, images, and voice anytime, anywhere by pressing your finger. This is the highlight of machine translation, something professional translators cannot achieve. Machine translation currently cannot understand and experience a specific culture through language and is not sensitive to culture. Different cultures have unique and different language systems, and machines do not have the complexity to understand or recognize slang, jargon, puns, and idioms. Therefore, machine-translated text may not conform to cultural values and specific norms, which is one of the challenges that machines need to overcome.

The breakthrough of artificial intelligence technology has greatly improved the effect of mechanical translation. Mechanical translation has gradually replaced artificial language translation, but mechanical translation of English-Chinese scientific and technological literature is not ideal. The construction of the neural network language model increases the intraword structure modeling and merging layer to form a new neural network language model [27, 28]. It provides the possibility to improve the effect of machine translation of scientific and technological literature in English and Chinese.

Few Chinese scientific and technological workers are proficient in English, and they encounter great obstacles in acquiring English-language scientific and technological literature. Moreover, native English speakers rarely master Chinese, which also limits their understanding of the progress of Chinese science and technology and affects academic exchanges.

Many studies have shown that machine translation models using deep learning technology have significantly improved the effect of translation, but obtaining a large number of parallel corpora in English and Chinese in the field of science and technology is the key to improving the translation effect of translation models. The lack of Chinese-English parallel corpora in the field of science and technology is the biggest weakness of current machine translation model training. The English-Chinese monolingual corpus can be obtained through published science and technology papers, and semi-supervised learning is introduced to make up for the lack of parallel corpora in English-Chinese machine learning for science and technology majors. Weakly parallel corpora do not have as strict alignment requirements as parallel corpora. The editor is relatively easy to edit and construct weakly parallel corpora and it introduces multidimensional methods to obtain English-Chinese parallel corpora to solve machine learning problems [29, 30].

In the mechanical translation training based on deep learning, in order to understand the translation process, the computer needs to transform the processed text into digital language. This process needs a word embedding operation. The main methods are one-hot representation and distributed representation. In one-hot representation, the length of the dictionary is consistent with the dimension of word embedding. For example, for the first word in the dictionary, its word is embedded as the first dimension, the value is 1, and the other dimensions are 0. In machine translation, we are faced with the problem of a large dictionary scale. The dimension of this expression method is too large and there is a problem of data scarcity.

Distributed representation can make up for the shortage of one-hot representation and integrate semantic information into word embedding. The model learns the sequence probability function and the distribution of words. Neural probability language can solve the problem of dimension, but the calculation of the training model is complex, which has an impact on the training effect of the whole model. In view of the shortcomings of neural network language models, many researchers have proposed a variety of training methods to improve the word embedding representation of the model, such as Word2vec. In order to convert sentences into embedded words, some experts proposed a CBOW (continuous bag of words) model based on target word context prediction, as shown in Figure 1.

Word embedding operations are the foundation of neural machine translation. Neural machine translation is an end-to-end translation method that relies on deep neural network structures in deep learning to translate one natural language into another. The transformer model is a neural machine translation model with better translation effect at present. The encoder-decoder of this model does not use the traditional inherent mode that must be combined with a convolutional neural network or a recurrent neural network, but only uses a multihead self-attention mechanism and a fully connected feedforward neural network.

The ransformer model still adopts the encoder-decoder architecture in structure, which is composed of multiple encoders and multiple decoders stacked. The encoder of the transformer model encodes the source language sequence (*x*_1_, *x*_2_,…, *x*_*n*_) into a hidden sequence of *z* = (*z*_1_, *z*_2_,…, *z*_*n*_). Then, we input *z* into the decoder and decode it into the output sequence (*y*_1_, *y*_2_,…, *y*_*n*_). Each step of the model is autoregressive [31]. When generating the next sequence at the decoder side, the previously generated sequence needs to be taken as the input of the decoder side and input to the decoder to participate in the calculation together.

The encoder contains two arithmetic modules. The first operation module is a multihead attention layer and the second operation module is a fully connected feed forward layer network module. Residual connections and layer normalization (Add & Norm) operations are used between the two modules [32, 33]. The structure of the decoder is similar to that of the encoder, the difference is that each block contains three operation modules, namely, the multihead self-attention module, the encoding-decoding self-attention module, and the fully connected feed forward network module.

### 3.2. Construction of a Deep Neurolinguistic Model

Neural machine translation (NMT) is an end-to-end translation system that completely uses neural networks to complete source language to target language translation [34]. The encoder-decoder framework is a classic framework for neural machine translation models, which can be implemented by different neural networks. In general, the input sentence from the encoder end to the source end generates semantic vectors layer by layer from low layers to high layers. The output of the last layer of the encoder and the hidden layer representation of the words that have been decoded are used as the input of the decoder. The decoding end obtains the translation corresponding to the target end through a series of calculations.

The transformer model only relies on the attention mechanism to complete the translation from the source language to the target language, and it is the model with a good effect at present. This model was proposed by Vaswani et al. [35], which belongs to the encoder-decoder structure, and the connection between the encoder and the decoder is realized through the attention mechanism. The encoder side and decoder side of transformer are, respectively, composed of *N* layers of the same network layer. Each layer of the encoder side includes two sublayers, a multihead self-attention mechanism, and a fully connected feedforward network layer. Residual connections and layer normalization are performed on the output of each sublayer. Similar to the encoder side, each layer of the decoder side includes an encoder-decoder attention sublayer in addition to the self-attention mechanism layer and the fully connected network layer. Likewise, residual connections and layer normalization are performed on the output of each sublayer at the decoder side.

English is the most commonly used language for people to communicate in the world and Chinese is the language that applies to the largest number of people. Due to the abundant English and Chinese corpus resources, great progress has been made in English-Chinese machine translation research, and the translation effect is good. Google Translate, Baidu Translate, etc. have adopted the neural network model [36]. Neural machine translation such as Google and Baidu usually rely on a large number of parallel sentence pairs to train translation models. At present, the Chinese and English data used for neural network model training are mainly concentrated in news, policy, and other fields. Due to the lack of parallel corpus data in the field of marine science and technology, Chinese-English machine translation does not perform well in the field of marine science and technology, and the translation results are unsatisfactory. The English-Chinese corpus in the field of marine science and technology is highly specialized. This paper intends to establish an English-Chinese corpus in the field of marine science and technology to improve the effect of machine translation of scientific and technological literature in this field.

We select 55 marine science and technology academic journals published in China (including fishery, petroleum, engineering and other marine-related publications), such as “Pacific Journal,” “Marine Fisheries,” “ Marine Geology & Quaternary Geology,” etc. The Chinese and English abstracts and partial full texts of all papers published from 1978 to 2022 were obtained through the database. We searched English papers related to marine science and technology in Web of Science database by keywords and selected English abstracts and some full texts. The Chinese and English abstracts collected from Chinese journals, in which Chinese and English sentences correspond, constitute the Chinese-English parallel corpus A, which has about 100,000 Chinese and English parallel sentence pairs. The translation model is trained with the Chinese-English parallel corpus A to obtain the initial translation model. Part of the Chinese full-text monolingual corpus collected by Chinese journals is translated into English by the initial translation model to generate an English monolingual corpus. The English monolingual corpus sentences translated by the machine and the input Chinese monolingual corpus sentences are spliced to form a synthesized bilingual corpus. Similarly, the full-text monolingual corpus of English papers collected in the Web of Science database is translated into Chinese through the initial translation model to generate a Chinese monolingual corpus. The Chinese monolingual corpus sentences translated by the machine are spliced with the input English monolingual corpus sentences to form a synthesized bilingual corpus. Through the above reverse translation technology, a large number of pseudo-corpora are generated and the Chinese-English enhanced corpus B is obtained. There are about 100,000 Chinese-English parallel sentence pairs in B, thereby expanding the corpus in the field of marine science and technology. The purpose of reducing data sparsity, improving model robustness, and improving translation effect is achieved. Finally, the parallel corpus A and the pseudo-corpus B obtained from the reverse translation are mixed in proportion to train the Chinese-English marine science and technology machine translation model. The data collection is shown in Figure 2 and the training of the translation model is shown in Figure 3.

In the attention mechanism, a query is embedded into the target retrieval response mapping function, and the specific calculation formula is shown below:

(1) $$\begin{array}{c} A\left(Q,K,V\right)=\text{soft}\max\left(QK^{T}\right)V. \end{array}$$

In (1), *A* (*Q*, *K*, *V*) represents the calculated attention value, Softmax expressed as a normalization function. In the transformer's attention network structure, the normalized function is used to process the attention weight as shown below:.

(2) $$\begin{array}{c} DA\left(Q,K,V\right)=\text{softmax}\left(\frac{QK^{T}}{\sqrt{d_{qk}}}\right). \end{array}$$

(2) *DA* (*Q*, *K*, *V*) expressed as zoom point attention, *Q*, *K*, *V* expressed as query embedded value, and $\sqrt{d_{qk}}$ represents a query embedded dimension.

In the multihead attention structure, we refer to the idea of ensemble as shown below:

(3) $$\begin{array}{c} {\text{head}}_{i}=DA\left(QW_{i}^{Q},KW_{i}^{K},VW_{i}^{V}\right). \end{array}$$

In (3), *QW*_*i*_^*Q*^, *KW*_*i*_^*K*^, *VW*_*i*_^*V*^ are trainable parameters.

(4) $$\begin{array}{c} \text{MHA}\left(Q,K,V\right)=\text{con}\tan\;t\left({\text{head}}_{1},{\text{head}}_{2},\ldots \ldots {\text{head}}_{h}\right) \end{array}$$

In (4), con tan *t* ( ) represents the concatenation operation of the embedding, *h* represents the number of head in the multi-head attention structure, and heads represents the *s*-th head.

In the transformer model, the encoder adopts the multi head attention mechanism and adds the feed forward neural network layer, and contains the output of two linear transformations and a ReLU activation function. The calculation of the activation function output is as follows:

(5) $$\begin{array}{c} FFN\left(x\right)=\max\left(0,xW_{1}+b_{1}\right)W_{2}+b_{2}. \end{array}$$

In (5), *W*_1_ and *W*_2_ are represented as weight matrices, and *b*_1_ and *b*_2_ are offsets, which are both model-trainable parameters.

In the model, word order information processing is shown by (6) and (7).

(6) $$\begin{array}{c} PE\left(\text{pos},2i\right)=\sin\left(\frac{\text{pos}}{10000^{2i/dm}}\right), \end{array}$$

(7) $$\begin{array}{c} PE\left(\text{pos},2i+1\right)=\cos\left(\frac{\text{pos}}{10000^{2i/dm}}\right). \end{array}$$

In (6) and (7), pos expressed as location information, *i* is the ordinal number of embedded words, and dm is the ordinal number of embedded words.

In order to better ensure that the word embedding layer of English-Chinese translation model has a good initial effect, we should first train the English-Chinese word embedding representation obtained by preprocessing and adopt self-learning method to express Chinese and English embedded words as *x* and *y*, Chinese and English words are embedded, and the rows and columns are, respectively, expressed as *x*′ and *y*′, At the same time, the linear transformation matrix is introduced to update the English-Chinese dictionary through the embedding operation of training mapping. Model training is carried out based on English-Chinese parallel corpus, in which (8) English-Chinese machine translation model training target formula.

(8) $$\begin{array}{c} L_{mt}\left(\theta \right)=E_{x^{\prime }∼D^{\prime },y^{\prime }∼D^{\prime }}\left[\left(-\log\;P_{x⟶y}\left(y^{\prime }|x^{\prime }\right)\right)+\left(\;-\log\;P_{y⟶x}\left(x^{\prime }|y^{\prime }\right)\right)\right]. \end{array}$$

In (8), *P*_*x*⟶*y*_ and *P*_*y*⟶*x*_ represent the translation model and *D* is the initial dictionary.

After the model is initialized, the whole model is trained based on the joint training method. In each training iteration, noise reduction code training will be carried out with English-Chinese weak parallel corpus, followed by English-Chinese and Chinese-English mutual translation training, and finally the translation model will be updated iteratively through English-Chinese translation loss. We maximize the relevance of H-line words in English-Chinese dictionary, as shown below:

(9) $$\begin{array}{c} \arg_{W_{x}W_{y}}\max\sum_{i}\sum_{j}D_{ij}\left(\left(X_{i}\cdot W_{X}\right)\cdot \left(Y_{j}\cdot W_{Y}\right)\right). \end{array}$$

In (9), the row of English word embedding represents *X*_*i*_, the column of Chinese word embedding represents *Y*_*j*_, and *W*_*x*_ and *W*_*y*_ are linear transformation matrices.

If *j* = arg_k_max(*X*_*i*_·*W*_*X*_)·(*Y*_*j*_·*W*_*Y*_), have *D*_*ij*_ = 1, otherwise *D*_*ij*_ = 0, The bilingual dictionary *D* is initialized, and the self-learning iteratively updates the dictionary *D* until convergence.

The overall training target formula of the machine translation model is shown below:

(10) $$\begin{array}{c} L_{\text{model}}\left(\theta \right)=\lambda_{ae}L_{ae}+\left(1-\alpha \right)\lambda_{mt}L_{mt}. \end{array}$$

In (10), *λ*_*ae*_ Model training loss ratio, *λ*_*mt*_ represents the loss ratio of translation training.

(11) $$\begin{array}{c} \lambda_{ae}=\left\{\begin{array}{cc} 0.5-\frac{\text{global\_step}}{\text{steps}}, & \text{ globa\_step}\leq \text{steps,}\\ 0, & {\text{global}}_{\text{step}}>steps. \end{array}\right. \end{array}$$

In (11) global_step is expressed as the current global steps of training.

### 3.3. Machine Translation Model Based on Local Weight Sharing and Encoder Fusion Output

Different languages have both substantive and formal commonalities. The former refers to the common components, structures, and rules of various languages, while the latter refers to the restrictions on grammatical rules and the description of rule forms. Implication commonness and nonimplication commonness. The former connects the emergence of certain language features with the emergence of other language features. If there is a fricative, there must be a stop, and if there is a front round lip vowel, there must be a back-round lip vowel. The latter can judge the existence of some language features without referring to other features. For example, each language has the difference between vowels and consonants. In addition, different languages also have absolute commonalities and tendency commonalities. The former refers to the commonness of all languages with and without exceptions, while the latter refers to the commonness existing as a tendency but with exceptions. There are both similarities and differences in the conversion between different languages. In the machine translation model, the common characteristics of different languages can be used to enhance the coding ability of the model, so as to improve the effect of language translation conversion.

In the bidirectional machine translation model of Marine Technology English-Chinese translation, transformer encoder submodule and transformer decoder submodule are adopted, respectively. At the same time, there are multiple structures of the same network in the encoder module. The English-Chinese machine translation model based on parallel corpus can learn more word meaning knowledge and optimize the initial value of the model through corpus training. However, in bidirectional machine translation between Chinese and English, there are two symmetrical groups of encoders and decoders, one for Chinese-to-English translation and the other for English-to-Chinese translation. Such a structure will lead to the repetition of model training parameters, increase the difficulty of training, and reduce the training effect, and there may be fitting problems in model training [12]. According to the cultural commonality, grammar, syllables, and other common characteristics of English and Chinese [24], the encoder module of the machine translation model is improved on the basis of local weight sharing and encoder sublayer fusion output to reduce the training parameters and improve the training effect.

The sublayers of the Chinese encoder and English encoder in this paper share weights (as shown in Figure 4). That is, the initial shared weight parameter values are the same, and the shared weight parameter values are updated simultaneously during the iteration process of the machine translation model training. As a result, the parameters of the machine translation model training are reduced, the difficulty of training is reduced, the training efficiency is improved, and the overfitting phenomenon in the model training process is alleviated.

The transformer model completely abandons the traditional recurrent neural network and convolutional neural network, improves the parallel computing ability, speeds up the training speed, and also makes the model lose the ability to capture local features. The output of the last sublayer of the transformer model encoder, as the output of the encoder, is input to the decoder. In this paper, the output information of the 6 sublayers of the encoder is fused as the output of the encoder and input to the decoder (as shown in Figure 4). In order to improve the information flow relationship between sublayers and sublayers, strengthen the ability of the encoder multilayer neural network to capture information, and improve the performance of NMT.

The outputs of each sublayer of the transformer model encoder are weighted and summed to form a new output, which is then input to each sublayer of the Transformer model decoder for decoding. In this way, the source language information output by each encoder sublayer is fully considered, so that the decoder can more fully capture the lexical, syntactic, semantic, and other information of the source language, and improve the translation effect. The weights for the weighted summation are obtained by training the models together.

Figure 4 shows the marine science and technology English-Chinese bidirectional translation model (MECM) with local weight sharing and encoder sublayer fusion output.

The model is mainly based on the transformer model structure of self-attention mechanism. The constructed English-Chinese dictionary is used to initialize the word embedding layer. Combined with the idea of local weight sharing, the weights of the first five layers of the model compilation module are set as shared coding, and the sixth layer uses its own English coding and Chinese coding. The mechanical translation decoder adopts its own decoder. At the same time, the weight sharing English-Chinese neuro mechanical translation model adopts the original joint training form, and the model training completes multiple rounds of iterative training. BLEU (Bilingual evaluation understudy) and semantic perplexity (PPL) are used as performance evaluation indicators. BLEU can evaluate the match rate of machine translated translations and reference translations, the higher the value, the higher the accuracy of machine translation. PPL evaluation can evaluate whether the translation results are smooth. The lower the value, the better. BLEU is calculated as shown below:

(12) $$\begin{array}{c} \text{BLUE}=BP\times \;\exp\left(\sum_{n=1}^{N}w_{n}\log\;p_{n}\right). \end{array}$$

In (12), w_n_ corresponding weight, *p*_*n*_ expressed as probability, *N* is the order, and the size is preset to 4, *BP* expressed as weight, The calculation formula is shown below:

(13) $$\begin{array}{c} BP=\left\{\begin{array}{cc} e^{1-r/t}, & t<r\\ 1, & t\geq r. \end{array}\right. \end{array}$$

In equation (13), *r* represents the length of the reference translation and *t* is the length of the translation translated by the machine.

*The PPLL* expression formula of evaluation index is shown below:.

(14) $$\begin{array}{c} PPL\left(S\right)=P{\left(w_{1}w_{2}\ldots \ldots w_{N}\right)}^{-1/N}. \end{array}$$

In (14), *S* represents the sentence, *N* represents the length of the sentence, and *P* (*w*_*i*_) is the probability that the order *i* word in the sentence *S* appears.

## 4. Data Testing of the Machine Translation Model Based on Deep Learning

The experimental data come from Chinese and English abstracts of Chinese and English academic journals related to marine science and technology, and there are a total of 7500 Chinese and English sentence pairs. Before the experiment, the dataset needs to be unordered, and then, the data are preprocessed. In order to ensure the feasibility of the English-Chinese machine translation model comparison experiment, the experimental environment remains unchanged [37]. At the same time, the encoder and decoder of the model are based on the standard transformer, and both use 6 encoder sublayers and 6 decoder layers. Moreover, we set the word embedding layer dimension, multihead attention layer dimension, feedforward network layer dimension, hidden layer dimension, and full connection layer dimension to 512, 8, 2048, 512, and 2048, respectively [38]. The model training adopts the Adam optimization area for updating optimization, and the internal optimizer parameter is set as the learning rate of 0.0001. In the model training, the over fitting problem should be avoided, and the parameter probability parameter will be set to 0.1 through dropout in the whole training.

The setting environment of the English-Chinese translation model with shared local weights involved in the comparison is the same. The number of encoders and decoders of the transformer is 6, but the first 5 submodules of the encoder will be set to be shared, and other parameters are the same as those of the Chinese translation model. The learning rate size is set to 2. Similarly, in order to avoid over fitting problems in model training, dropout will be passed in the whole training and its parameter probability parameter will be set to 0.1.

In the English-Chinese machine translation model test of marine science and technology based on parallel corpus, the two submodels used are analyzed and tested, the word embedding layer of the experimental model is randomly initialized, and noise reduction self-encoding operation is carried out. For the modeling of the English-Chinese parallel corpus model of marine science and technology, the word embedding layer of dictionary initialization is still adopted, but the noise reduction self-encoding operation is removed, and the corresponding loss parameter is set to 0. The whole experimental test environment is consistent, and the BLEU value is introduced into the evaluation standard. The Chinese and English abstract sentence pairs of Chinese marine scientific papers are selected as test samples, and the number of samples is 7500. The English abstract sentences of Chinese marine science and technology journals are used as artificial translations, and the corresponding Chinese abstract sentences are input into the network, and the output is the translated sentence translated by the machine, and the BLUE value is calculated accordingly. At the same time, we select 3 models from Google Translate, Bing Translate, Baidu Translate, Youdao Translator, and Lingos Translator, and denote them as *A*, *B*, and *C*, respectively. We translate 200 samples and calculate the BLEU value to evaluate the translation effect of the software.

Figure 5 is a comparison of the test results of different translation models. It can be seen that in the aspect of English-Chinese bidirectional translation, the MECM model using local weight sharing and encoder sublayer fusion output has the highest BLEU value. Compared with the transformer model, the BLEU of the MECM model is improved by 1.6 (Chinese-English) and 3.8 (English-Chinese), respectively. The BLEU of the MECM (-fusion) model with local weight sharing and without encoder sublayer fusion output is improved by 1.2 (Chinese-English) and 1.7 (English-Chinese), respectively. The BLEU of the MECM (-Fusion) model without local weight sharing and with encoder sublayer fusion output improves by 0.8 (Chinese-English) and 0.8 (English-Chinese), respectively. The MECM model combining local weight sharing and encoder sublayer fusion output achieves better translation results. Models that only use local weight sharing, or only use encoder sub-layer fusion output models, also have a certain improvement in translation effect.

The comparison of the test results of different models and translation software is shown in Figure 6. From the comparison of BLEU values in the English-Chinese and Chinese-English translation directions in Figure 6, it can be found that the translation software *A*, *B*, and *C* are not as effective as the MECM model and the transformer translation model. The best performing software A among the translation software, its BLEU values are 3.4 (Chinese-English) and 6.1 (English-Chinese) lower than those of the MECM model, and 1.8 (Chinese-English) and 2.3 (English-Chinese) lower than those of the transformer model. The difference in the translation effect is obvious. The BLEU value of the best performing software A among the translation software is 11.5 (Chinese-English) and 8.2 (English-Chinese) higher than that of the worst performing software C, which is a significant difference. This is because the MECM model and the transformer model are trained using marine science and technology-related corpora, which are of the same type as the tested samples, which improves the translation quality. Although the translation software A, B, and C also use deep learning neural networks, their training samples are relatively broad and their professionalism is not strong, so the translation effect for marine science and technology texts is not good. There are also significant differences in the performance of translation software A, B, and C, which may be related to the translation technology and training data they use.

Using the marine science and technology English-Chinese corpus and test data, the performance of the transformer model and the marine science and technology English-Chinese model MECM are tested.  Figure 7 shows the relationship between the number of iteration steps of the two models and the BLEU value. From the comparison of the BLEU values of the English-Chinese and Chinese-English translation directions of the marine science and technology text in Figure 7, it can be found that the effect of the marine science and technology English-Chinese model MECM is better than that of the transformer model. For Chinese-English and English-Chinese translations, the BLEU values of the MECM model after convergence are 1.14 and 2.94 higher than those of the transformer model, respectively. For the Chinese-to-English model, the transformer model is trained in 220 steps to converge, while the MECM model only needs to be trained for 180 steps. The two models translated from English to Chinese have similar rules.

We use the test set data selected from the marine science and technology literature to evaluate the translation results of the MECM translation model in this paper and use the semantic PPL (perplexity) as the performance evaluation index; the result is shown in Figure 8.

As can be seen from Figure 8, in the MECM translation model in this paper, the PPL of the marine science and technology literature test set decreased by 91.53% and 91.09% in the English-Chinese translation and Chinese-English translation processes, respectively. The lower the PPL value, the higher the fluency of the sentence, which also shows that the idea of local weight sharing and encoder sublayer fusion output can be applied to the translation model to achieve better translation results.

In the training of the marine science English-Chinese translation model MECM based on local weight sharing, the number of shared layers of the encoder was changed to test the effect of the number of shared layers on the BLEU value. The model in which the encoders share *X* layers (*X* = 1, 2, 3, 4, 5, 6) is represented as MECM (*X*), such as MECM (5), which means that the encoders share 5 layers. The test results are shown in Figure 9.

As can be seen from Figure 9, the BLEU values of the English-Chinese bidirectional translation of the MECM model are significantly higher than those of the transformer model. Therefore, it can be concluded that the English-Chinese machine translation model of marine scientific and technological documents with local weight sharing has better translation effect. The BLEU value of the MECM model with the encoder sharing 5 layers is the largest, so the encoder sharing 5 layers can achieve better translation effect. This paper adopts the encoder sharing 5-layer MECM model.

The PPL value was used to test and evaluate the MECM model, transformer model and translation software, and the results are shown in Figure 10.

As can be seen from Figure 10, in the performance test of semantic confusion index, the PPL value of the Chinese-English bidirectional translation model is lower than that of the translation software. The PPL value of the MECM model is lower than that of the transformer model, and the PPL values of the Chinese-English and English-Chinese translation directions drop by 18.72% and 14.62%, respectively. The lower the PPL value, the higher the fluency of the sentence, indicating that the idea of local shared weights and the fusion output of the encoder sublayer can be applied to the translation model to achieve better translation effects. The PPL value of translation software A is comparable to that of the transformer model, indicating that translation software A also shows better translation fluency. The performance of translation software B and C is not good and needs to be further improved.

## 5. Conclusion

This paper uses the existing neural network technology to train the existing English-Chinese machine translation. Based on deep learning technology, we collect Chinese and English abstracts and partial full texts of Chinese and English papers with marine science and technology as the key words and build a professional corpus in English and Chinese about marine science and technology. In the Chinese-English bidirectional translation model, the local weight sharing is introduced into the Chinese encoder and the English encoder, and the output of the Chinese encoder sublayer and the English encoder sublayer is fused as the output of the respective encoders, and the performance of the translation model is evaluated using the BLEU parameters. Through the training of the translation model, compared with the transformer model, the BLEU value of the model with local weight sharing and encoder sublayer fusion output is improved by 1.6 and 3.8 in the Chinese-English and English-Chinese translation directions, respectively. The PPL values in the Chinese-English and English-Chinese translation directions decreased by 18.72% and 14.62%, respectively. Experiments show that the research of machine language adaptive technology based on deep learning can more smoothly realize the English-Chinese bidirectional translation of marine scientific and technological literature. On the basis of traditional machine translation, a translation model based on deep neural algorithm is proposed, and a professional Chinese and English material library is obtained through the database, which improves the effect of model training. However, this paper does not analyze the model efficiency of translation in different languages, there are certain limitations, and this part needs further research.

## Figures and Tables

**Figure 1:** CBOW model structure diagram.

**Figure 2:** Schematic diagram of data collection.

**Figure 3:** Schematic diagram of translation model training.

**Figure 4:** Marine science and technology English-Chinese bidirectional translation model (MECM) with local weight sharing and encoder sublayer fusion output.

**Figure 5:** Comparison of test results of different models.

**Figure 6:** Comparative experimental results of different models on the test.

**Figure 7:** Relationship between iteration steps of different models and BLEU value. (a) Chinese-English translation. (b) English-Chinese translation.

**Figure 8:** PPL trend chart of the language model.

**Figure 9:** Comparative experimental results of different models on the test.

**Figure 10:** PPL values for models and translation software.

## Data Availability

The data used to support the findings of this study are included within the article.

## References

[1] Chakravarthi B. R., Rani P., Arcan M., McCrae J. P. (2021). A survey of orthographic information in machine translation. *SN computer science*.

[2] Brown P. F., Cocke J., Pietra V. J. D. (1990). A statistical approach to machine translation. *Computational Linguistics*.

[3] Liu S., Li C. H., Zhou M. Statistic machine translation boosted with spurious word deletion[C].

[4] Kharb S., Kumar H., Kumar M., Chaturvedi A. K. Efficiency of a machine translation system.

[5] He X., Deng L., Rose R., Huang M., Trancoso I., Zhang C. (2020). Introduction to the special issue on deep learning for multi-modal intelligence across speech, language, vision, and heterogeneous signals. *IEEE Journal of Selected Topics in Signal Processing*.

[6] Bonsignorio F., Hsu D., Johnson-Roberson M., Kober J. (2020). Deep learning and machine learning in robotics [from the guest editors]. *IEEE Robotics and Automation Magazine*.

[7] Tripathi S., Sarkhel J. K. (2010). Approaches to machine translation [J]. *Annals of Library and Information Studies*.

[8] Charoenpornsawat P., Sornlertlamvanich V., Charoenporn T. Improving translation quality of rule-based machine translation.

[9] Stahlberg F. (2020). Neural machine translation: a review. *Journal of Artificial Intelligence Research*.

[10] Ye Y. P. (2021). Translation mechanism of neural machine algorithm for online English resources. *Complexity*.

[11] Laskar S. R., Paul B., Paudwal S., Gautam P., Biswas N., Pakray P. Multimodal neural machine translation for English-Assamese pair.

[12] Zhang X. Research on machine translation and computer aided translation based on cloud computing.

[13] Li J. X., Wang P. T. (2022). Research on transfer learning-based English-Chinese machine translation. *Mobile Information Systems*.

[14] Zhang J. C., Luan H. B., Sun M., Zhai F., Xu J., Liu Y. (2021). Neural machine translation with explicit phrase alignment. *IEEE/ACM Transactions on Audio, Speech, and Language Processing*.

[15] Sennrich R., Haddow B., Birch A. Improving neural machine translation models with monolingual data[C].

[16] Poncelas A., Popovic M., Shterionov D. S., Wenniger G. M. D. B. Combining SMT and NMT back-translated data for efficient NMT [C].

[17] Imankulova A., Dabre R., Fujita A., Imamura K. (2019). Exploitingout-of domain parallel data through multilingual transfer learning for low-resource neural machine translation [C]. *Proceedings of machine translation summit XVII*.

[18] Wu J. W., Wang X., Wang W. Y. Extract and edit: an alternative to back-translation for unsupervised neural machine translation [C].

[19] Currey A., Heafield K. Zero-resource neural machine translation with monolingual pivot data [C].

[20] Chen K. H., Wang R., Sumita E. (2022). Integrating prior translation knowledge into neural machine translation. *IEEE/ACM Transactions on Audio, Speech, and Language Processing*.

[21] Lin L., Liu J., Zhang X., Liang X. (2021). Automatic translation of spoken English based on improved machine learning algorithm. *Journal of Intelligent and Fuzzy Systems*.

[22] Ercan G., Haziyev F. (2019). Synset expansion on translation graph for automatic wordnet construction. *Information Processing & Management*.

[23] Lora M., Vinco S., Fummi F. (2019). Translation, abstraction and integration for effective smart system design. *IEEE Transactions on Computers*.

[24] Dhanjal A. S., Singh W. (2021). An automatic machine translation system for multi-lingual speech to Indian sign language. *Multimedia Tools and Applications*.

[25] Chauhan S., Daniel P. (2022). A comprehensive survey on various fully automatic machine translation evaluation metrics. *Neural Processing Letters*.

[26] Liu X. J. (2022). Evaluation of the Accuracy of Artificial Intelligence Translation Based on Deep Learning. *MOBILE INFORMATION SYSTEMS*.

[27] Wu L., Wu L. (2021). Research on business English translation framework based on speech recognition and wireless communication. *Mobile Information Systems*.

[28] Dai X., Yin H., Jha N. K. (2020). Grow and prune compact, fast, and accurate LSTMs. *IEEE Transactions on Computers*.

[29] Ba Y., Qi L. (2021). Construction of WeChat mobile teaching platform in the reform of physical education teaching strategy based on deep neural network. *Mobile Information Systems*.

[30] Song G. (2021). Accuracy analysis of Japanese machine translation based on machine learning and image feature retrieval. *Journal of Intelligent and Fuzzy Systems*.

[31] Graves A. (2013). Generating sequences with recurrent neural networks. https://arxiv.org/abs/1308.0850.

[32] Lei J., Ryan Kiros J., Hinton G. E. (2016). Layer normalization. https://arxiv.org/abs/1607.06450.

[33] Gehring J., Auli M., Grangier D., Yarats D., Dauphin Y. N. Convolutional sequence to sequence learning [C].

[34] Shi X., Ning Q., May J., Knight K. (2021). Enhancing information transfer in neural machine translation [J]. *Computer Engineering & Science*.

[35] Vaswani A., Shazeer N., Parmar N. Attention is all you need[C].

[36] An B., Long C. J. (2022). Paraphrase based data augmentation for Chinese-English medical machine translation [J]. *Journal of Electronics and Information Technology*.

[37] Kocmi T., Federmann C., Grundkiewicz R., Junczys-Dowmunt M., Matsushita H., Menezes A. (2021). To Ship or Not to Ship: An Extensive Evaluation of Automatic Metrics for Machine Translation [J]. https://arxiv.org/abs/2107.10821.

[38] Ban H., Ning J. (2021). Design of English automatic translation system based on machine intelligent translation and secure Internet of things. *Mobile Information Systems*.

